The article "Cardiac Arrest following a Myocardial Infarction in a Child Treated with Methylphenidate" was retracted in 2021. Reasons: errors in the analysis; errors in the results or conclusions; unreliable results or conclusions.

# Cardiac Arrest following a Myocardial Infarction in a Child Treated with Methylphenidate

**DOI:** 10.1155/2015/905097

**Published:** 2015-06-28

**Authors:** Kim Munk, Lise Gormsen, Won Yong Kim, Niels Holmark Andersen

**Affiliations:** ^1^Department of Cardiology, Aarhus University Hospital, Palle Juul-Jensens Boulevard 99, 8200 Aarhus N, Denmark; ^2^Department of Psychiatry, Aarhus University Hospital, Risskov Skovagervej 2, 8240 Risskov, Denmark

## Abstract

The use of psychostimulants labeled to treat attention deficit/hyperactivity disorder increases. Among side effects these drugs raise blood pressure and heart rate, and the safety has been scrutinised in recent years. Data from large epidemiological studies, including over a million person-years, did not report any cases of myocardial infarction in current users of methylphenidate, and the risk of serious adverse cardiac events was not found to be increased. We present a case with an 11-year-old child, treated with methylphenidate, who suffered cardiac arrest and was diagnosed with a remote myocardial infarction. This demonstrates that myocardial infarction can happen due to methylphenidate exposure in a cardiac healthy child, without cardiovascular risk factors.

## 1. Introduction

The risk of cardiovascular events and sudden death related to attention deficit/hyperactivity disorder (ADHD) medications has been scrutinized in the recent years [1–5].

In adults, the initiation of methylphenidate has been found to be associated with nearly a doubling of the rate of sudden death or ventricular arrhythmia [3]. However, in children and adolescents, large scale population studies have not found an increased cardiovascular risk in ADHD drug users [1]. Although one study reported a high hazard ratio estimate for “sudden death or ventricular arrhythmia” with methylphenidate use, the results were nonsignificant [4].

In children and adolescents, a low absolute number of cardiovascular events may explain why hazard ratios, even in large scale studies, come out nonsignificant. However, with the reported spreads in confidence intervals, one cannot rule out the possibility of an increase by as much as a tripling of the risk for serious cardiovascular events.

Mechanisms behind cardiovascular disease and methylphenidate are not fully understood. Methylphenidate increases heart rate, increases blood pressure, and potentially causes arterial vasospasms, due to the increased levels of circulating catecholamines [5, 6]. All these factors could theoretically increase cardiovascular risk [5]. There are no valid data to suggest that methylphenidate directly increases the corrected QT interval or induces arrhythmia [5, 7].

We present a case with a child treated with methylphenidate that suffered from cardiac arrest during exercise and was diagnosed with a remote myocardial infarction.

## 2. Case Presentation

The patient is an 11-year-old boy with attention deficit/hyperactivity disorder and Tourette syndrome. Two years prior to the current incident he had been seen by a pediatric psychiatrist over a course of time and was finally treated with methylphenidate. He was slowly uptitrated to the maximum appropriate dose of 54 mg per day (36 + 18 mg per day/body weight 50 kg), which had been ongoing ever since.

Apparently, the child had been feeling well, but a week before his admission he felt dizzy and light headed after vigorous trampoline jumping. His mother noticed he had tachycardia but thought nothing of it. The incident only lasted a few minutes and afterwards he was well.

On the day of admission, the patient had been in conflict with one of his peers. To calm down, the patient was sent to the gym court, to exercise and play ball. After a few minutes he left the court and fell down with cardiac arrest due to ventricular fibrillation. He was successfully resuscitated by school staff and the prehospital service.

Upon hospital arrival the child was sedated and intubated. He was circulatory stable and he was treated with hypothermia for 24 hours. A urine toxicology screening only showed traces of the anesthetics used during the resuscitation and methylphenidate according to the prescribed dose.

Both the initial ECG and the ECGs after hypothermia (Figure 1) showed Q-waves in leads I, AVL, and V4–6 and ventricular ectopic beats. The QT intervals were normal. The echocardiogram did not show any congenital defects but impaired left ventricular function due to regional wall motion abnormalities and thinning of the myocardial wall, consistent with a previous myocardial infarction in the circumflex artery area. There was only a minor increase in the troponin levels, which could be explained by the cardiac arrest, and the initial infection parameters were normal.

A coronary computed tomography angiography scan showed normal coronary artery anatomy with a dominant left coronary artery and no signs of myocardial bridging. However, a subsequent cardiac magnetic resonance scan showed clear signs of an old myocardial infarction with delayed hyperenhancement and thinning of the lateral wall of the left ventricle, corresponding to the circumflex artery supply (Figure 2).

To exclude paradox emboli, a transesophageal echocardiogram with bubble contrast was done. No atrial septal defects or mural thrombi were found. A full panel of blood coagulation tests did not reveal any coagulation disorder or hypercholesterolemia.

Before discharge, a coronary angiogram was done, which confirmed the computed tomography angiography result but also excluded abnormal coronary spasm tendency by a methylergometrine test. The patient also had an invasive electrophysiology study, which showed normal atrioventricular conduction without accessory pathways and an easily inducible sustained ventricular tachycardia, deriving from the scar tissue in the left ventricle. Subsequently, an implantable cardioverter defibrillator was implanted, and the patient was put on a low dose of metoprolol succiante (25 mg), with a treatment plan to increase the dose at a later stage. The methylphenidate treatment was discontinued. A wide panel of genetic disorders related to tachyarrhythmia was examined, which all came out negative.

Three weeks after discharge the child was on his own in a bouncy castle on a Friday evening. After 15 minutes of exercise, he shortly felt ill and sat down but recovered quickly without any recollection of chest pain or any other discomfort. The following Monday, the defibrillator telemetry showed that the pacemaker had defibrillated an episode of ventricular fibrillation (Figure 3). Following this episode, the metoprolol succiante dosage was increased to 100 mg o.d. over two weeks.

## 3. Discussion

Acute myocardial infarction due to atherosclerotic plaque rupture is a leading cause of death and disability. However, in childhood and adolescence, myocardial infarction is extremely rare and other causes should be sought such as coronary artery anomalies, vasculitis, and coagulation defects. Due to the extremely rare occurrence in children, a myocardial infarction diagnosis may not be suspected and therefore overlooked. Likewise, myocardial infarction in children treated with methylphenidate is extremely rare. In two large epidemiological studies, including over half a million person-years of follow-up, of current users of attention deficit/hyperactivity disorder medications, not a single myocardial infarction was reported during treatment [1, 4]. The boy in this case report presented with cardiac arrest without any prior complaints about chest discomfort or shortness of breath. The only symptom was the short exertion induced tachycardia episode a week before the major event. Had this been presented for a physician, it is unlikely that it would have led to further diagnostic workup. In retrospect this episode was most likely caused by ventricular tachycardia.

The large epidemiological studies on methylphenidate are based on reported diagnoses, among which this boy's myocardial infarction diagnosis probably would never have appeared. Instead, he suffered from cardiac arrest and would have been classified as sudden cardiac death, had he not been resuscitated.

When the boy was admitted, the first assumption was a primary arrhythmia. However the ECG clearly indicated regional myocardial necrosis and the echocardiogram showed thinning of the myocardial wall. The CMR scan clearly indicated that the myocardial infarction was of an older date (more than weeks) due to thinning of the myocardium and an adversely remodeled left ventricle.

Currently there is no recommendation in Denmark or by the FDA to obtain ECG before and during methylphenidate treatment, explaining why there was no ECG prior to treatment. Theoretically, there may be more children with undiagnosed myocardial infarctions among methylphenidate users that are missed, if routine ECGs are not obtained on a regular basis. In the present case, the Q-waves in the ECG would have disclosed that the child had developed heart disease. Whether this would have altered the course is speculative.

Obviously it may be questioned if the myocardial infarction actually developed prior to methylphenidate treatment and if it really was the cause. It is now two years since the index admission. The boys present clinical situation is quite concerning. Despite high dose ACE-inhibitors and beta-blockers his left ventricle has further adversely remodeled from an initial internal diastolic diameter of 5.4 cm to 7.2 cm on the latest echocardiography. His ejection fraction has deteriorated to 35%. He is in heart failure class II. He recently underwent two VT ablations due to long lasting tachycardia episodes and therapies from the ICD. Therefore it is unbelievable that this boy was started on methylphenidate after the huge myocardial infarct. He would have been in overt heart failure which would have been noticed. Children do not develop huge myocardial infarcts without a cause. This young boy has been very thoroughly examined. He did not suffer from hypertension or hypercholesterolemia, and there was no coronary artery anomaly, no myocardial bridging, no coagulation defects, no PFO, and no abnormal coronary spasm tendency to explain his myocardial infarct. Furthermore, the dosage of methylphenidate was uptitrated correctly to an appropriate dosage and there was not any suspicion of abuse. The only thing that points out is the methylphenidate treatment, which FDA recognizes can cause heart attacks in adults.

Randomized trials show that ADHD drugs reduce symptoms significantly, compared to placebo [8], and improve children's learning and academic achievement modestly [9]. At present, the use of ADHD drugs is increasing. For this reason, even though registry studies do not show associations with cardiovascular events in children, it is important to closely monitor and report cardiovascular events to ensure that this treatment remains well controlled, efficient, and safe.

In conclusion, myocardial infarction and sudden cardiac death are extremely rare among children during treatment with methylphenidate. However, the present case shows that myocardial infarction can happen due to methylphenidate exposure in a cardiac healthy child, without any other cardiovascular risk factor.

## Figures and Tables

**Figure 1:** 12-lead electrocardiogram obtained on day five of the index admission. Abnormal Q-waves are seen in the left sided leads I, aVL, and V4–V6. The QTc interval was normal at 395 msec (Fredericia correction).

**Figure 2:** Cardiac magnetic resonance (CMR) imaging showing short-axis views in diastole (a) by cine CMR and (b) by late gadolinium enhancement imaging. Arrows indicate myocardial wall thinning and late gadolinium enhancement in the circumflex artery area consistent with myocardial necrosis and scar formation.

**Figure 3:** Reading from the implantable cardioverter defibrillator showing onset of ventricular fibrillation (arrow) at an average cycle length of 210 ms corresponding to a rate of 285 per minute. After the first shock (HV) delivered by the defibrillator, sinus rhythm is restored.
